# Magnetic Resonance Images, Pathological Features of Thrombus, and Expression of NLRP Inflammasome in Patients with Acute Ischemic Stroke

**DOI:** 10.1155/2022/3464042

**Published:** 2022-08-16

**Authors:** Xiaoqin Wang, Wenhui Kou, Weidan Kong, Shujing Ma, Qian Xue, Yuan Zou, Aixia Song

**Affiliations:** Department of Neurology, The First Affiliated Hospital of Hebei North University, Zhangjiakou 075000, Hebei, China

## Abstract

The aim of this study was to investigate imaging features of magnetic resonance imaging (MRI), pathological features of thrombus, and expression of nucleotide-binding oligomerization domain-like receptors protein 3 (NLRP3) inflammasome in acute ischemic stroke (AIS). Their relationship with the prognosis of patients was also explored. Sixty patients with AIS admitted to the hospital were selected as the observation group, and 20 healthy objects were in the control group. The shape of the thrombus was observed by MRI, pathological features of the thrombus were observed under hematoxylin-eosin (HE) staining, and the levels of NLRP3 inflammasome and inflammatory factors in serum were detected. The MRI-T2 weighted imaging (T2WI) signal ratio and plaque enhancement rate in the observation group were higher than those in the control group significantly (*P* < 0.05). In the observation group, the red/mixed thrombus in 6–12 h and 24 h were also much higher than that in 6 h (*P* < 0.05). The levels of NLRP3, interleukin-1*β* (IL-1*β*), interleukin-18 (IL-18), and tumor necrosis factor-*α* (TNF-*α*) in the observation group were higher than those in the control group in 6 h, 6–12 h, and 24 h (*P* < 0.05), and those reached the highest levels in 24 h. The ratio of fibrins/platelets in the cardiogenic thrombus reached (63.8 ± 15.6) %, which was significantly higher than that in the large-artery atherosclerotic thrombus (49.5 ± 14.2) %, *P* < 0.05. The ratio of red blood cells (RBCs) in the large atherosclerotic thrombus was (30.7 ± 14.3) %, considerably lower than (42.9 ± 15.2) %, *P* < 0.05. The prognosis of patients with the fibrin/platelet-rich thrombus was highly lower than that with the RBC-rich thrombus (*P* < 0.05). The levels with poor prognosis were higher than those with good prognosis (*P* < 0.05). MRI could be used to assist in the assessment of brain conditions in patients with AIS. NLRP3 inflammasome was involved in the inflammatory response of AIS and can be used for predicting the poor prognosis, having a certain clinical application value. In addition, different types of thrombi also laid a certain impact on prognosis.

## 1. Introduction

Acute ischemic stroke (AIS) is clinically referred to as cerebral infarction, which is the occlusion of cerebral arteries that leads to infarction in cerebral tissues, accompanied by damage to some nervous system functions. Its onset is rapid with complex and variable pathogenesis, not only causing physical harm to the patients but also bringing about a heavy mental burden psychologically [1]. The key to timely treatment of AIS patients is to open the occluded blood vessels as soon as possible, restore blood flow as quickly as possible, and save the brain tissues in the ischemic penumbra. The better the reconstruction of blood flow, the better the prognosis of patients. In clinical treatment, clinical symptoms can be improved by drug therapy and rehabilitation therapy [2]. With the development of imaging technology, magnetic resonance imaging (MRI) is widely used in the diagnosis and treatment of clinical diseases [3, 4]. Intravenous thrombolysis and emergency mechanical thrombectomy (MT) within the time window recommended by current guidelines are the most effective treatments for AIS. However, the current narrow time window and low recanalization rate greatly limit the application of intravenous thrombolysis, and the prognosis of patients with MT varies greatly depending on the etiology and time [5].

Previous studies have found that the composition and size of the thrombus are closely related to the recanalization rate of intravenous thrombolysis and the difficulty of MT. Therefore, an in-depth understanding of the pathological features of thrombosis may bring new strategies for the diagnosis and treatment of AIS [6]. Most of the previous studies about the pathology of AIS thrombosis were carried out by imaging, serology, autopsy pathology, and other methods. With the widespread application of emergency MT, the fresh cerebral arterial thrombus can be taken out through MT. Thereby, the composition, type, and features over time of the thrombus can be analyzed, and the relationship with prognosis further can also be studied by combining with the different etiologies of patients' occlusion as well as other clinical data [7].

As the main cause of AIS, especially large-scale cerebral infarction, intracranial and extracranial atherosclerosis have a very complex formation mechanism. In 2002, Tschopp's team first discovered that inflammasomes play an important role in it. Nucleotide-binding oligomerization domain-like receptors protein 3 (NLRP3) is the core of inflammasome, and its activation and activity regulation are of important physiological and pathological significance in the process of atherosclerosis [8]. Previous studies have proved that NLRP3 may be involved in the formation of coronary atherosclerosis as an inflammasome. In this research, hematoxylin-eosin (HE) staining and immunohistochemistry were performed on the thrombus obtained by MT in patients with AIS, and the control thrombus was prepared to analyze the basic components of the thrombus and the expression of NLRP3 in patients with AIS and then to discuss the correlation among them [9]. Although a large number of studies have suggested that intravenous thrombolysis and MT have marked benefits for patients with AIS, and their effective rate is poor due to varied etiologies and time [10, 11]. In this research, the composition, etiology, features, interaction with neuro-vessels, and inflammatory factors in the thrombus in AIS patients were observed and analyzed. Utilizing the information, a more comprehensive understanding can be gained of the interaction of the thrombus and drugs, thrombectomy stents, as well as the vessel wall. Thus, it can enable clinicians to predict the thrombosis situation more accurately and then formulate more accurate treatment plans, benefiting more patients. The information may offer new hope for future treatment of AIS. All in all, this work brought new hope for the treatment of AIS in the future, by observing and analyzing the composition, etiology, features, and inflammatory factors in the thrombus of AIS patients.

## 2. Materials and Methods

### 2.1. Research Objects

Sixty patients with AIS were included in the observation group, as they were admitted to the hospital during the period from January 2018 to December 2020. These research objects selected met the following inclusion and exclusion criteria. In the control group, 20 healthy objects met the above exclusion criteria. The 20 cases in the control group were healthy people who met the exclusion criteria. No abnormalities were found in their cranial computerized tomography (CT)/MRI, magnetic resonance angiography (MRA), and cervical artery color Doppler ultrasound. Compared with the observation group, the control group showed no significant difference in the age and gender of objects (*P* > 0.05). This research had been approved by the ethics committee of the hospital, and the included patients as well as their families signed the consent forms.

#### 2.1.1. Inclusion Criteria

(1) The patients were 18–85 years old. (2) In view of anterior circulation, MT and angioplasty were performed within 8 hours of onset. For posterior circulation, it could be extended to within 24 hours of onset, MT for progressive stroke was guided by imaging, and the treatment time was prolonged as appropriate. (3) In the clinical diagnosis of AIS, symptoms and focal neurological impairment were corresponding to the suspected occluded vascular innervation area. Meanwhile, the symptoms and signs of neurological damage did not relieve for more than 60 minutes. (4) The score of the National Institutes of Health Stroke Scale (NIHSS) for neurological impairment was >6 points, and the score of Alberta Stroke Program Early Computerized Tomography (ASPECT) was ≥6 points. (5) In imaging evaluation, intracranial hemorrhage was excluded through CT. CT angiography (CTA) or MRA examination of the head and neck confirmed that the occluded blood vessel was the internal carotid artery or vertebral basilar artery, and there was a certain amount of collateral circulation compensation.

#### 2.1.2. Exclusion Criteria

(1) The time window of MT was exceeded. (2) Cranial CT showed cerebral hemorrhage or large-area cerebral infarction, as the volume of cerebral infarction exceeded 1/3 of the cerebral hemisphere (anterior circulation) or 1/3 of the brainstem (posterior circulation). (3) They underwent active bleeding or a major surgery within the past two weeks; they used to have significant trauma or bleeding disease. (4) They were allergic to contrast media. (5) The score of the modified Rankin Scale (mRS) was >3 points before onset. (6) They had the bleeding constitution or were receiving anticoagulation therapy, including coagulation factor deficiency and the international normalized ratio (INR) > 1.7. (7) They got refractory hypertension that cannot be controlled by drugs (systolic blood pressure ≥185 mm·Hg or diastolic blood pressure ≥110 mm·Hg), the blood glucose <2.8 mmol/L or >22.0 mol/L, and the platelet count <100 × 10^9^/L. (8) They suffered from severe liver or kidney dysfunction. (9) Their life expectancy was less than three months. (10) They disagreed to sign the informed consent forms.

### 2.2. Imaging Examination

A 3.0T superconducting scanner was used for MRI scanning. The scanning parameters were set, including the time of echo (TE) 1.9 ms, time of repetition (TR) 3.0 ms, T1 6.8 ms, matrix 256 × 256, slice thickness 6 mm, and interval 1 mm. The transverse and coronal planes of patients were scanned and analyzed with the aid of contrast agents. Dynamic enhanced scanning was also made on patients, and the results were interpreted and summarized by a professional radiologist.

### 2.3. Evaluation Indicators

The clinical data of 60 patients were analyzed retrospectively. Apart from the name, age, and gender, their medical history of hypertension, diabetes, hyperlipidemia, cerebral infarction, and myocardial infarction; their history of taking antiplatelet drugs or anticoagulant drugs; as well as their history of smoking and drinking were also investigated. Others for analysis included the Trial of ORG 10172 in Acute Stroke Treatment (TOAST) etiology classification, diseased blood vessels, size, and location of the thrombus as well. For the time from onset to vascular opening, whether intravenous thrombolysis was performed before MT, the times of MT, and whether stents were used, were observed. Complications, the NIHSS score after 24 hours and 3 months, the mRS score, and others were included likewise.

The obtained fresh thrombus was fixed in 4% paraformaldehyde solution, transferred to 70% ethanol solution within 48 hours, embedded in paraffin, and sectioned serially to make paraffin sections with a thickness of 3 *μ*m. The samples were stained with HE staining solution, and the HE staining characteristics were observed with an optical microscope.

5 mL of fasting venous blood was collected from each object in the observation group and the control group. After anticoagulant treatment and centrifugation, serum was obtained. As the instructions of the enzyme-linked immunosorbent assay (ELISA) kit were followed, the levels of NLRP3 inflammasome and inflammatory factors, such as interleukin-1*β* (IL-1*β*), interleukin-18 (IL-18), as well as tumor necrosis factor-*α* (TNF-*α*), in serum were detected.

### 2.4. Statistical Analysis

SPSS 22.0 was applied for statistical processing, as the measurement data were expressed as ($\bar{x}$ ± *s*). The *t*-test was adopted for comparison between the two groups, one-way analysis of variance was for the comparisons among two groups, and the paired *t*-test was for changes in different time periods in the observation group. The enumeration data were analyzed using the *χ*^2^ test. *P* < 0.05 indicated a statistically significant difference.

## 3. Results

### 3.1. Comparison of General Data of Objects

The general data were analyzed between the observation group and the control group. As could be found from Table 1, there was not a significant difference in age, gender, body mass index (BMI), history of hypertension, history of diabetes, history of myocardial infarction, history of smoking, and history of drinking between the observation group and the control group (*P* > 0.05). The number of patients with a history of hyperlipidemia and cerebral infarction was higher in the observation group than those in the control group, showing significant differences statistically (*P* < 0.05).

### 3.2. MRI Features of AIS Patients

The comparison of MRI features between the observation group and the control group was displayed in Figure 1. There were obvious structural changes in the cerebral MRI images of patients in the observation group, among which the diffusion-weighted imaging (DWI) features were the most obvious. From the quantitative comparisons in MRI parameters shown in Figure 2 between the observation group and the control group, the T2 weighted imaging (T2WI) signal ratio and plaque enhancement rate of the observation group were higher than those of the control group, with big differences statistically (*P* < 0.05).

### 3.3. Pathological Features of Thrombosis in Patients with AIS

First, HE-stained sections were made for the analysis of pathological features of the thrombus in AIS patients in the observation group, as the results were presented in Figure 3. According to the vascular components, the thrombus of the patients was mainly divided into a red thrombus (Figure 3(a)), white thrombus (Figure 3(b)), and mixed thrombus (Figure 3(c)). The white thrombus was mainly composed of a large number of platelets and a small amount of fibrin, while the red/mixed thrombus consisted of a large amount of fibrin, red blood cells (RBC), and a small number of platelets.

Then, the pathological features of the thrombus were compared within the observation group for 6 h (25 cases), 6–12 h (29 cases), and 24 h (6 cases), as shown in Figure 4. With the increase in onset time, the proportion of patients with the red/mixed thrombus also increased remarkably. The proportion of the red/mixed thrombus in 6–12 h and 24 h was higher than that in 6 h, with the difference being statistically significant (*P* < 0.05).

### 3.4. Expression of Inflammation-Related Indicators in Patients with AIS

The levels of NLRP3, IL-1*β*, IL-18, and TNF-*α* were compared between the two groups in different time periods. As shown in Figure 5, the levels of NLRP3, IL-1*β*, IL-18, and TNF-*α* in the observation group were notably higher than those in the control group, with statistically significant differences (*P* < 0.05). In the observation group, the levels of NLRP3, IL-1*β*, IL-18, and TNF-*α* in 6–12 h and 24 h were greatly higher than those in 6 h, and the differences were also significant statistically (*P* < 0.05). The levels of IL-18 and TNF-*α* were much higher in 24 h than in 6–12 h, suggesting significant differences statistically as well (*P* < 0.05).

### 3.5. Expression of Inflammation-Related Indicators in AIS Patients with Different Prognoses

The levels of NLRP3, IL-1*β*, IL-18, and TNF-*α* were compared between the observation subgroups with different prognoses. From Figure 6, the levels of NLRP3, IL-1*β*, IL-18, and TNF-*α* of the poor prognosis group were markedly higher than those of the good prognosis group, with significant differences statistically (*P* < 0.05).

### 3.6. TOAST Classification of Thrombus Components from Different Sources and Their Correlations with Prognosis

Among the different sources of TOAST classification, the proportion of fibrins/platelets in the cardiogenic thrombus was (63.8 ± 15.6) %, which was greatly higher than the (49.5 ± 14.2) % of large-artery atherosclerotic thrombus, *P* < 0.05. The proportion of RBCs (30.7 ± 14.3) % was notably lower than (42.9 ± 15.2) % in the large-artery atherosclerotic thrombus, *P* < 0.05. There was a little difference in the content of white blood cells between the two types of thrombi from different sources (*P* > 0.05). In the 3-month mRS score for a good prognosis rate, the prognosis of patients with the white thrombus was remarkably lower than that of patients with the red thrombus, *P* < 0.05, with the statistically significant difference shown in Figure 7.

## 4. Discussion

MRI can detect early small lesions and exclude intracranial hemorrhage and other diseases; it is helpful for clinicians to evaluate the neurological impairment of patients and is of great significance to the early diagnosis, treatment, and prognosis of patients [12, 13]. The advantage of MRI in diagnosing AIS lies in that it is a multi-directional imaging technique so that small lesions can be observed in hard-to-find areas such as the brainstem. It eliminates the interference of bone artifacts and reduces the misdiagnosis rate [14]. Timely assessment and treatment could be given to reduce infarct size, restore normal blood supply around the infarction, and reduce the impact of infarction on surrounding organs. Reduction of the damage to brain tissue caused by long-term ischemia and hypoxia can restore normal neurological functions of patients [15]. Under DWI technology, old and new infarcts can be clearly distinguished, thereby diagnosing the diseases and reducing the missed diagnosis rate of such diseases [16]. Therefore, for patients with suspected AIS and no other contraindications, DWI sequence scanning should be conducted as soon as possible. In this work, MRI was applied for analyzing the changes in cerebral features of patients with AIS, which were also compared with those of healthy people. The MRI-T2WI and dynamic-contrast enhanced MRI images could show the infarct location clearly. Endovascular treatment of AIS enables routine pathological examination of cerebral arterial thrombosis. The current studies found that the pathological features of the acute cerebral arterial occlusive thrombus were similar to postmortem pathological examinations [17]. Whether from the heart or arteries, the thrombi have similar structural features and cannot simply be classified as a red or white thrombus.

Studies have shown that with the reduction of the thrombus, NLRP3 and its activation of related downstream cascade responses declined [18]. To this end, the levels of NLRP3 and its downstream inflammatory factors IL-18, IL-1*β*, as well as TNF-*α*, were compared and analyzed between AIS patients and healthy people in different time periods. The results of this work indicated that the levels of NLRP3, IL-18, IL-1*β*, and TNF-*α* in patients with AIS in different time periods were extraordinarily higher than those in healthy people. This suggested that NLRP3 and related downstream signaling pathways were activated in patients with AIS, consistent with the findings of previous studies. With the disease development of AIS patients, the levels of NLRP3, IL-18, IL-1*β*, and TNF-*α* became increasing gradually in 6 h, 6–12 h, and 24 h. Thus, NLRP3 and related downstream signaling pathways could be progressively increased or activated with the development of AIS. Some studies have shown that the NLRP3 inflammasome in peripheral blood can help the oxidation of low-density lipoprotein and lipid peroxidation directly, inducing a significant increase in the generation of free oxygen radicals. Then, endothelial cells will be damaged, resulting in the release of endothelin and inflammatory factors, accelerating the formation of atherosclerosis, and finally leading to stroke [19]. Other studies have confirmed that the NLRP3 inflammasome in peripheral blood can activate platelets in vivo, promote platelet adhesion and aggregation, and then cause thrombosis [20]. For further exploration of the correlation between NLRP3 and the prognosis of AIS patients, the changes in NLRP3, IL-18, IL-1*β*, and TNF-*α* levels were analyzed in AIS patients with different prognoses. The levels of NLRP3, IL-18, IL-1*β*, and TNF-*α* in the good prognosis group were distinctly lower than those in the poor prognosis group. It was suggested that the activation of NLRP3 and its downstream inflammation-related signaling pathways would affect the prognosis of patients with AIS and result in a poor prognosis.

The main components of a thrombus include fibrins/platelets, white blood cells, and RBCs. The results of this research proved that the proportion of fibrins/platelets in the cardiogenic thrombus was (63.8 ± 15.6) %, which was notably higher than (49.5 ± 14.2) % in the large-artery atherosclerotic thrombus, *P* < 0.05. The proportion of RBCs reached (30.7 ± 14.3) %, significantly lower than the (42.9 ± 15.2) % of the large-artery atherosclerotic thrombus, *P* < 0.05. There was not a significant difference in white blood cell content (*P* > 0.05). Some studies have shown that the ratio of fibrins/platelets in the cardiogenic thrombus is significantly higher than that in the noncardiogenic thrombus, and there are fewer RBCs [21]. In addition, the RBC-rich red thrombus has higher viscosity and variability as well as lower elasticity and stiffness, which can improve the success rate of thrombectomy in patients. The fibrin/platelet-rich white thrombus has a higher friction coefficient than the red thrombus [22], increasing the difficulty of thrombectomy. The prolonged recanalization time of occluded blood vessels will lead to prolonged ischemia of brain tissues and then affect the clinical prognosis of patients. It was suggested from the research results that in the good prognosis rate of the mRS score at 3 months, the prognosis of patients with the fibrin/platelet-rich white thrombus was significantly lower than that with the RBC-rich red thrombus, *P* < 0.05.

## 5. Conclusion

MRI-T2WI of patients with AIS showed high-signal features, and MRI-DWI could display the cerebral infarction location of patients clearly. As AIS developed, the levels of NLRP3, IL-18, IL-1*β*, and TNF-*α* showed a trend of gradual increase, and those levels in patients with poor prognosis also increased notably. It was indicated that NLRP3 as well as its downstream inflammation-related signaling pathways were involved in the process of AIS and affected the prognosis of patients. In addition, different types of thrombi also affected the prognosis of patients. This research had certain limitations. The sample size was relatively small, and no animal model was prepared for the further verification of the inevitable connection between NLRP3 activation and the accelerated progression of AIS. Therefore, more in-depth research in this direction was expected to be carried out in the future.

## Figures and Tables

**Figure 1:** Comparison of MRI features between the two groups.

**Figure 2:** Comparison of MRI quantitative parameters between the observation group and the control group. (a) Signal ratio of T1WI; (b) signal ratio of T2WI; (c) plaque enhancement rate. ^*∗*^Compare with the control group, *P* < 0.05.

**Figure 3:** HE staining observation of the thrombus in the observation group (×400). (a) Red thrombus; (b) white thrombus; (c) mixed thrombus.

**Figure 4:** Pathological type distribution of the thrombus in the observation group. ^*∗*^Compared with those in 6 h, the differences were of statistical significance, with *P* < 0.05.

**Figure 5:** Comparison of levels of serum-related indicators between the two groups. (a) NLRP3; (b) IL-18; (c) IL-1*β*; (d) TNF-*α*. ^*∗*^, ^#^Compared with the corresponding results of the control group, 6 h observation group, and 6–12 h observation group, respectively, *P* < 0.05.

**Figure 6:** Comparison of serum-related indicator levels in the observation group with different prognoses. (a) NLRP3; (b) IL-18; (c) IL-1*β*; (d) TNF-*α*. ^*∗*^Compared with those of the good prognosis group, *P* < 0.05.

**Figure 7:** The correlation between thrombus components from different sources in TOAST classification and the mRS score. ^*∗*^Compared with the cardiogenic thrombus, *P* < 0.05. ^#^Compared with the patients with rich RBCs, *P* < 0.05.

**Table 1:** Comparative analysis of general data between the two groups.

Data	Observation group (60 cases)	Control group (20 cases)	*P* value
Male (*n* (%))	33 (55.0)	12 (60.0)	0.667
Age (years old)	61.2 ± 5.9	60.3 ± 4.2	0.343
BMI (kg/m^2^)	25.3 ± 2.8	26.1 ± 2.6	0.418
History of hypertension (*n* (%))	34 (56.7)	9 (45.0)	0.134
History of diabetes (*n* (%))	22 (36.7)	6 (30.0)	0.409
History of hyperlipidemia (*n* (%))	37 (61.7)	8 (40.0)	0.033
History of cerebral infarction (*n* (%))	15 (25.0)	1 (5.0)	0.016
History of myocardial infarction (*n* (%))	7 (11.7)	2 (11.0)	0.547
History of smoking (*n* (%))	33 (55.0)	11 (55.0)	0.889
History of drinking (*n* (%))	26 (43.4)	6 (30.0)	0.416
Cardiogenic thrombus (*n* (%))	36 (60.0)	—	—
Large-artery atherosclerotic thrombus (*n* (%))	24 (40.0)	—	—

## Data Availability

The data used to support the findings of this study are available from the corresponding author upon request.
